The article "Developments and Clinical Applications of Biomimetic Tissue Regeneration using 3D Bioprinting Technique" was published in 2022. Journal: Appl Bionics Biomech.

# Developments and Clinical Applications of Biomimetic Tissue Regeneration using 3D Bioprinting Technique

**DOI:** 10.1155/2022/2260216

**Published:** 2022-12-20

**Authors:** Hamza Abu Owida

**Affiliations:** Medical Engineering Department, Faculty of Engineering, Al-Ahliyya Amman University, Amman 19328, Jordan

## Abstract

Tissue engineers have made great strides in the past decade thanks to the advent of three-dimensional (3D) bioprinting technology, which has allowed them to create highly customized biological structures with precise geometric design ability, allowing us to close the gap between manufactured and natural tissues. In this work, we first survey the state-of-the-art methods, cells, and materials for 3D bioprinting. The modern uses of this method in tissue engineering are then briefly discussed. Following this, the main benefits of 3D bioprinting in tissue engineering are outlined in depth, including the ability to rapidly prototype the individualized structure and the ability to engineer with a highly controllable microenvironment. Finally, we offer some predictions for the future of 3D bioprinting in the field of tissue engineering.

## 1. Introduction

Tissue engineering has been employed in therapeutic settings to get around the shortage of donor organs. Ultimately, the goal of tissue engineering is to produce functional tissue that may be used to replace wounded tissue [1].

Tissue repair and regeneration in regenerative medicine have historically struggled due to a lack of appropriate techniques. Researchers are always trying to perfect artificial tissues that can replace natural ones in the hopes that they may be used one day in clinical practice [2].

Three-dimensional (3D) printing emerged as an additive manufacturing process in the last few decades, and it has since seen fast development in the field of regenerative medicine. With the advent of 3D bioprinting technology, we now have the chance to create artificial tissues that function and look much like natural ones [3]. With this method, cell-rich materials are layered in 3D structures using computer-aided design methodologies. Thanks to developments in fields like nanotechnology, cell biology, materials science, and engineering, 3D bioprinting is finding more and more uses in fields like tissue engineering [3, 4]. There are currently three technologies utilized for 3D bioprinting: inkjet bioprinting, extrusion bioprinting, and laser-based bioprinting. The main benefit of using 3D bioprinting in tissue engineering is that it allows for the hierarchical and spatial distribution of cells, hydrogels, and active substances according to the intended 3D functionality. Cultured cell adhesion, development, cell signaling, and gas and transmits of nutrients are all facilitated by the porous, networked nature of 3D-bioprinted materials. When compared to more conventional methods, this can help tissue regeneration quite a long bit [4–7]. In addition, a significant number of findings based on 3D bioprinting have been published occur annually (Figure 1).

The bioprinting technology employed in tissue engineering is the primary subject of this review. This article elaborates on the large variety of tissues for which bioprinting can be used to fabricate tissue, highlighting its role in tissue regeneration. Additionally, the possibility, challenges, and advantages of creating a framework for tissue regeneration are highlighted. In this article, we will discuss the various applications of 3D bioprinting in tissue repair.

## 2. Bioprinting Technologies

The growing field of 3D bioprinting uses computer simulations to accurately prescribe the building of a 3D living cell system in vitro. The method is akin to fast prototyping or additive manufacturing in that it involves building a tissue or organ in layers [1, 4].

Multiple 3D printing methods have matured since their inception. Microextrusion molding, laser sintering, and stereolithographic have replaced inkjet printing as the dominant manufacturing technique. The most popular types of 3D printing will be discussed in detail below (Figure 2).

### 2.1. Inkjet-Based 3D Bioprinting

Several droplet sheets can be printed using an inkjet printer to make 3D models. Small amounts of low-viscosity bioink (1–100 pl) are deposited onto the substrate by inkjet during hydrogel 3D printing [8]. Of these methods, thermal-induction inkjet printing involves heating liquid droplets with a thermal actuator before expelling them from the print head at high speed. Inkjet printing's deposition method may successfully mold the material into the desired form (Figure 3). The solution may be delivered to the nozzle in precise amounts, which is a distinct advantage. However, this approach has some limitations, such as the requirement that the biological components used be in liquid droplet form. The second challenge is that there is a maximum material viscosity for inkjet printers [8–10].

### 2.2. Microextrusion 3D Bioprinting

Hydrogel filaments are deposited onto a surface via nozzles in microextrusion bioprinting, which make use of a software diffusion system that employs needles, valves, or hydraulic pressures. For extrusion bioprinting to work, the bioink utilized must be highly viscous and cross-linkable so that the printed object retains its 3D shape (Figure 4). Extrusion bioprinting provides several advantages over other 3D printing methods, including greater printing precision, a faster printing speed, and the ability to print with a wider range of materials. Extrusion printing technology has one distinct benefit over inkjet bioprinting: it can employ a broader range of bioinks. Therefore, extrusion printing is the prevalent technique for tissue bioprinting. Cells are dehydrated and lack nutrition after printing and the printing precision is restricted, and the static friction of the sheet cells' survival capacity could be affected by substances on the jet exterior [1, 4, 11].

### 2.3. Laser 3D Bioprinting

Pulsed laser beams are used in the process of laser-based bioprinting. This causes differential pressure, which in turn pushes the base material cells from the original printing medium “ribbon” onto the receipt materials. Due to a lack of nozzle, laser-assisted bioprinting never experiences technical problems related to nozzles, and neither is the damage and death of cells caused by shear stress, which can occur once the size of the jet is very tiny and the bioink has an excessive viscosity; therefore, this method's compatibility with advantage from the organic substance's viscosity (Figure 5). High spatial resolution is a further advantage of laser-assisted bioprinting. Higher cell densities can be printed using this technology, allowing for more precise regulation of cell–cell interactions and a more detailed high-definition print. However, it is rarely used in tissue engineering because of the high cost of the necessary hardware and software [12, 13].

### 2.4. Stereolithographic-Based 3D Bioprinting

In order to deliberately cross-link bioinks using a process that involves layers, stereolithographic bioprinting makes use of ultraviolet light. By strategically directing UV light, we may exert unparalleled control over the cross-linking of macromolecules, thereby stimulating tissue formation (Figure 6). Stereolithographic printing has several benefits, including high resolution (100 m) and high cell survival (>85%). Like laser-based printing, this approach does not need a nozzle; hence, clogged nozzles are not an issue. Due to the strong photopolymerization ability required, however, only a select few bioinks may be employed. UV radiation, which is used in conventional stereolithographic bioprinting, can be damaging to cells and may trigger mutations. This issue has been resolved via novel bioink that can be cross-linked with illumination and cell attachment that significantly improves cell viability and has significant applications in the fields of bioprinting and tissue regeneration [14, 15].

### 2.5. Bioinks for 3D Bioprinting

Support structures materials, cultured cells, and bioactive molecules, given the vast quantity of printable organs and tissues, are all common components of bioink, the central component of 3D printing. Improved 3D printability and biocompatibility are only two of the many benefits offered by today's generation of bioinks. Shear thinning capabilities, found in interpenetrating networks, nanocomposites, and supramolecular hydrogels, for instance, allow them to bypass this barrier previously present in bioinks. These biological functions can be vastly improved by other developing inks, such as those containing functional groups and nanoparticles with biologically active capabilities [16, 17]. Nearly a hundred different kinds of modified biological materials are currently in use as bioinks.

### 2.6. Biomimetic Tissue Regeneration using 3D Bioprinting Technique

Restoration, maintenance, improvement, and replacement of various biological tissues are all possible through tissue engineering, which is the application of cells, engineering, materials technologies, and appropriate biochemical parameters. Applications for 3D bioprinting techniques with varying capabilities and characteristics in tissue engineering can be found across the medical spectrum [18].

#### 2.6.1. Bone Tissue

Bone tissue, which composes the bone of vertebrates, is a stiff organ that serves several functions, including providing protection for the body's internal organs, cell production, mineral storage, and so on. Bone is a form of hard tissue, which consists of dense connective tissue with an interior honeycomb-like matrix, making the bone stiffer. Hydrogel scaffolds have attracted a lot of attention because of the configurations available and the fact that their characterizations can be adjusted [19].

In order to create physically toughened and long-term steady photo-crosslinkable hydrogel scaffolds, Poldervaart et al. [20] modified the naturally natively hyaluronan with minimal loss of biocompatibility. Irradiating the hydrogels with ultraviolet radiation increased the power compressibility and Young's modulus, both of which noted growing hydrogel solidity. The biocompatibility experimental studies with bone hematopoietic stem cells mesenchymal stromal cells demonstrated that the custom-made scaffolds for 3D bioprinting could be made from polymathic hyaluronic acid hydrogel and therefore would aid in promoting bone growth.

After testing the efficacy of bioinks containing fibrous collagen gels alone versus bioinks containing serum stem cells, bone marrow-derived stem cells, and collagenous fibers for the treatment of wounds, the former group was found to be superior in terms of wound contraction and endothelial renewal. Microvessel density and capillary breadth grew more in amniotic fluid stem cell-treated wounds than in bone marrow stem cells. Healing and thrombosis may be due to cell-secreted nutrients, not cell-to-cell communication, observing the fluorescent dye cells after 14 days revealed that the bioprinted cells stayed in a switching cycle, implying that they were not indefinitely incorporated into the tissue [21].

Human mesenchymal stem cells' expansion and osseointegration were boosted by Tan et al.'s synergist's use of 3D bioprinting using ultrasonic pulses of short wavelength. Scaffolds with tailored architecture were printed using optical mediated stereolithography (SLA) bioprinters. In order to stimulate cell adhesion, growth, and proliferation, the results showed that the porous interconnecting scaffolds should be subjected to ultrasonic pulses of short wavelength at a frequency of 1.5 MHz and a duty cycle of 20%, with an intensity of 150 mW cm^2^. These unique approaches also confirmed the viability and efficacy of combining ultrasound with 3D bioprinting to enhance cell activity, particularly for orthogenesis in bioprinted scaffolds [18].

In order to improve surface interactions, research group created collagen hydrogels made of 2D nesosilicates, they are essentially nanomaterials with an extremely high percentage of heterogeneity and functioning despite their incredibly thin structure. Hydrogels containing nanosilicates enhanced osteogenic differentiation in the lack of any osteoinductive agent and had a compression elasticity that was four times higher than that of collagen-only hydrogels (Figure 7). The findings demonstrated that nesosilicates functioning as bioactive factors facilitated bone regeneration by increasing its strength properties and permeability, among other benefits [22].

A research group [23] developed image-guided bioamendment in approach using Pluronic F-127 cell shipper to boost cell survival and expedite osteogenesis of osseointegration mesenchymal stem cells with rhBMP4 in a hydrogel structure and the osteogenic differentiation. The results demonstrated that photo-biomodulation is a good candidate to guide and speed up bone tissue engineering.

#### 2.6.2. Cartilage Tissue

Cartilage is a connective tissue that does not have its own blood supply or central nervous system. Chondrocytes are a specialized sort of cell that can be found there. Matrix diffusion of nutrients is delayed since there are no blood arteries to carry the nutrients directly to the cells [24].

Recent study employed a mixture of hyaluronan hydrogel, which they then inserted under the skin of hairless rats. After multiple time points, the implant was subjected to histological, immunohistochemical, and mechanical analyses, compared to control studies, the implantation had good machinability, suggesting that cell and hydrogel mixtures could create like-cartilaginous tissue in vivo [25].

Nguyen et al. [26] turned to two bioinks: nanofibrillated cellulose containing alginate (NFC/A) and nanofibrillated cellulose containing hyaluronic acid with induced pluripotent stem cells (iPSC). After a set amount of time in culture, cartilage tissue was visible under the microscope, proving that the NFC/A bioink was superior for iPSC bioprinting and thus serving as a valuable resource for cartilage regeneration. Although alginate hydrogel was commonly used in earlier studies in terms of its suitability as an integrin substance, the material exhibited poor mechanical qualities due to its inherent great flexibility and brittleness.

Structural elements with high cell viability and robust mechanical qualities were investigated by Rhee et al. [27], who used collagen hydrogels with fibrochondrocytes to manufacture them. Human nasal chondrocytes were used in a nanofibrillated cellulose–alginate hydrogel carrier to create human ear-like constructions, these showed a high cell survival rate (86%) after 7 days of in vitro culture, proving that the nanocellulose-based bioink was suitable for 3D bioprinting. Studies demonstrated that nanocellulose-based hydrogels might be employed as support materials when creating live tissues, for example, Ávila et al. [28] combined nanocellulose–alginate-based hydrogels and human nasal chondrocytes to create ear cartilage analogs.

The combination of polypropylene glycol (PG) and HA in the bioink resulted in greater cell survival and differentiation compared to the bioink containing only PG. As a 3D scaffold material, graphene oxide (GO) has been employed to support regenerated cartilage and facilitate the transport of critical growth factors. The expression of collagen I in cartilage was considerably upregulated along the boundary between the tissue and a 3D-printed GO scaffold designed for the production of cartilage matrices [29].

#### 2.6.3. Skin Tissue

Human skin consists of several layers and is home to many different cell types and functional units, including sweat glands and blood arteries. The skin's primary role is to act as a sensory organ and a heat sink. When the skin sustains a mild, localized injury, the body can repair the wound on its own by producing keratin and fibrinogen, but in more severe cases, skin transplant is required [30].

Major skin injuries are common in everyday life, creating a global demand for skin tissue substitutes. By depositing keratinocytes, melanocytes, and fibroblasts and creating a suitable survivable milieu akin to genuine skin tissues, Ng et al. [31] were able to create a 3D-layered porous structure in vitro. These results demonstrated that the 3D-bioprinted skin texture, in contrast to the colored skin structure made by standard approaches, more closely resembled natural skin in aspects of the developed multilayered. By using a pneumatically controlled bioprinter, Lee et al. [32] demonstrated that human skin progenitors and epithelial tissue could be cultured in a biomimetic layered epidermis via 3D printing for possible skin repair. A similar in situ skin printer for repairing burn wounds was created by Seol et al. [33].

They used this skin printer to effectively distribute keratinocytes and fibroblasts to the injured areas of pig skin, and the results showed that the epithelium could regenerate and wounds could heal quickly. In a study of wound treatment, Skardal et al. [21] compared to a bioink containing solely fibrous collagen gels, the combined group healed wounds and regenerated epithelium at a much faster rate. Microcirculation integrity and microvascular dimension grew more in serum stem cell-treated wounds than bone marrow mesenchymal stem cell-treated lesions. After 2 weeks, fluorescently bioprinted prolong the lifetime transitory, indicating they were not fully incorporated into the tissue. This shows that wounds healing and vasculature are caused by cell nourishment, not cell-to-cell interaction.

Using the same two types of cells and a laser-assisted bioprinting approach, Michael et al. [34] developed a fully cellularized skin substitute that was evaluated in the dorsal skin fold chamber of hairless mice. Once the transplants were ready, they were inserted into full-thickness skin wounds and left there for 11 days. This demonstrated the successful 3D bioprinting of a cell construct by laser-bioprinting and the tissue development in vivo. The results demonstrated the feasibility of using laser-assisted bioprinting to create 3D multicellular structures.

Stereolithographic bioprinting was used by Zhu et al. [35] to create neural structures using mouse neural stem cells, gelatin methacrylamide hydrogels, and graphene nanoplatelets. After 2 weeks, neuronal differentiation and neurite outgrowth were observed in the bioprinted structures harboring neural stem cells, demonstrating their remarkable regenerative potential and inspiring novel ideas for the use of 3D bioprinting in the field of neuroscience.

#### 2.6.4. Neural Tissue

Bundled nerve fibers transport signals from one region of the body to another and carry out additional functions, such as healing damaged nerves and brain tissue. Spinal neuronal progenitor cells (sNPCs) and oligodendrocyte progenitor cells (OPCs) were produced from iPSCs, and the spinal cord was printed using extrusion-based multimaterial bioprinting (OPCs). Rebuilding operational nerve fibers interconnection throughout areas of primary nervous tissue injury can be helped by bioprinting OPCs in mixture with sNPCs. The findings showed the product's ability to construct biomimetic, hydrogel-based scaffolds imitating anatomical structures in vitro and for using these structures to create new strategies for addressing neurological illnesses [36, 37].

Stereolithographic bioprinting was used by Zhu et al. [35] to create neural structures using mouse neural stem cells, gelatin methacrylamide hydrogels, and graphene nanoplatelets. After 2 weeks, neuronal differentiation and neurite outgrowth were observed in the bioprinted structures harboring neural stem cells, demonstrating their remarkable regenerative potential and inspiring novel ideas for the use of 3D bioprinting in the field of neuroscience.

Lee et al. [38] showed that vascular endothelial growth factors (VEGFs) could be directly bioprinted and designed for slow release from a fibrin scaffold, proving the technique's viability. When compared to controls, VEGF-secretion-induced morphological alterations in implanted murine neural stem cells led to enhanced cell migration. Recently, Ilkhanizadeh et al. [39] showed that macromolecular gradients inside bioprinted scaffolds could be generated via inkjet printing to stimulate brain stem cell development. They added fetal growth factor 2 (FGF2), ciliary neurotrophic factor (CNTF), or fetal bovine serum (FBS) to the bioink made from polyacrylamide and studied its influence on primary fetal neural stem cells. While CNTF and FBS promoted the production of the astrocyte marker glial fibrillary acidic protein (GFAP) and the smooth muscle marker smooth muscle actin, respectively, in the presence of FGF2, the neural stem cells maintained their proliferative identity. Next, they made a scaffold with a gradient of CNTF concentrations from high to low and watched the cells differentiate along the gradient. More specifically, CNTF treatment resulted in elevated GFAP expression levels in the treated cells.

Dai et al. [40] have produced a tumor model by enclosing glioma stem cells in a gelatin/alginate/fibrinogen bioink to simulate the tumor extracellular matrix. This model was used to show that glioma stem cells had the ability to become blood vessels by displaying high levels of VEGF, a hallmark of tumor angiogenesis. In a subsequent study, Wang et al. [41] enhanced this work by developing a bioink made of alginate, gelatin, and glioma stem cells that mimics the glioma microenvironment and allows for the examination of tumor vascularization. Glioma stem cells were discovered to release vascular endothelial growth factor A and to form tubule-like structures in vitro when they were enclosed within the scaffold. After being transplanted into mice, glioma stem cells developed into blood arteries made up of tumor cells with an aberrant endothelium phenotype.

#### 2.6.5. Cardiovascular Tissue

A gelatin hydrogel was used in a unique way by Hasan et al. [42] to create multilayered blood arteries on a microfluidic device. It took the researchers only 3–5 days for the endothelial cells to mature and be properly positioned and grown within the vessel walls after they had been seeded and the physical structure of the vessels had been created. Similar results were seen by Bertassoni et al. [43] when they used agarose in a crosslinked hydrogel to print a blood artery and then grew it with endothelial cells. Others have looked into the possibility of using bioprinting to speed up the body's natural functions, in addition to the more straightforward method of direct implantation of bioprinted components (Figure 8). Gaebel et al. [44] bioprinted and implanted a cardiac patch cultivated with mesenchymal stem cells and endothelial cells into rat hearts with infarction. This preclinical investigation showed that 3D bioprinting might be used to enhance angiogenesis and aid in cardiac tissue recovery after myocardial infarction.

Using human cardiac cells and a hydrogel dubbed FRESH, Lee et al. [45] from Carnegie Mellon University successfully bioprinted a heart valve tissue. Cells were placed into the hydrogel and cultivated for an additional 28 days after the hydrogel was bioprinted on the support material by rapid pH change-driven gelation. Bioprinted valve tissue had a diameter of around 28 mm and a resolution of about 20 mm (the filament). With the wall thickness increased to 14% during contraction, the structure was able to contract synchronously and execute directional potential action propagation. In order to test the viability of 3D bioprinting in this context, Duan et al. [46] from Cornell University tried to employ a hybrid hydrogel made of hyaluronic acid and gelatin, mixed with human aortic valvular interstitial cells to build a trilobal valve catheter by extrusion bioprinting.

Using a combination approach based on extrusion bioprinting, Zhang et al. [47] created an endothelialized cardiac construct. Myocardial cells capable of spontaneous and synchronous contraction were generated by first forming a layer of fused endothelial scaffold and then implanting them on a 3D endothelial bed. Applications for endothelialized myocardial platforms include cardiovascular toxicity testing, drug discovery, and illness simulation.

Most recently, Liu et al. [48] used DLP bioprinting to shape neonatal mouse ventricular cardiomyocytes to create a cardiac microtissue in photo-crosslinkable hydrogels that mimics the microarchitecture and function of a normal ventricular myocardium. The in vitro model is capable of synchronized contractions and a forced output that is determined by the established benchmarks. According to the findings, the in vitro tailored cardiac tissue can be used as a platform for cardiac disease modeling and medication screening, thereby laying the groundwork for heart engineering.

Applications include drug screening and toxicity testing, as well as the prospect of building a human-sized working in vitro heart in the future, as shown by the results [49]. The valvular microtissues comprising porcine valvular interstitial cells were encapsulated in a sort of modified gelatin as the instructional material to create large-scale 3D microtissue using UV-light crosslinking, as demonstrated by Roosens et al. [50]. Using multicellular valvular microtissues as building blocks, we were able to generate the hypothesis that microchips may be assembled in such soft modified gelatin hydrogels using DLP or triphenylphosphine bioprinting technologies to construct functional, large-scale organoids. For their bioprinting work, Lee et al. added a second layer of bone marrow-derived mesenchymal stem cells (bMSCs) in sodium alginate on top of a diagonally cross-stripped polycaprolactone (PCL) scaffold. The second layer is then covered with a third, this time in a helical PCL scaffold. In our investigation of pulsatile flow's effect on bMSCs, we find that the cells undergo endothelial-like differentiation [51].

#### 2.6.6. Lung Tissue

Lungs are a crucial part of the respiratory system because they transfer oxygen from the air into the blood and carbon dioxide from the blood into the atmosphere. Lee et al. [51] from Rice University used SLA bioprinting and a biocompatible photocurable hydrogel to create a lung-like air sac. Several attempts to make the hydrogel absorb blue light and speed up the curing process were unsuccessful until a graduate student suggested using food coloring. The inside anatomy of the 3D-printed air sac was complex, including blood vessels and air passages. It was because of this architecture that the air sac was able to both provide oxygen to its environment and pump air into the airways. The lung model's size was comparable to a cent, and its resolution was 0–50 mm. Furthermore, the lung analog was sturdy enough to withstand breathing tests. Compared to more traditional methods, it may complete printing tasks in minutes rather than hours or days 35. Also, Tan et al. [18] created a small liver using primary stem cells and put it into mice with chronic liver damage. The fact that these liver cells were able to survive in vitro suggests that they might be able to do so in vivo as well, suggesting that the bioprinted blood arteries might be able to supply them with the nutrients they need to stay alive.

Huh [52] developed an in vitro lung-on-a-chip that reconstituted 3D microarchitecture, dynamic mechanical activity and integrated the physiological function of the alveolar–capillary interface. The physiological function of the alveolar–capillary interface was integrated into an in vitro “lung-on-a-chip,” which also reproduced 3D microarchitecture and dynamic mechanical activity. The goal was to simulate the physiological and mechanical properties of the space between the lungs and the rest of the body. A thin (E10 mm), porous, elastomeric polydimethylsiloxane (PDMS) membrane separates the upper and bottom cell culture chambers in the lung model. Human alveolar epithelial cells were seeded in the upper chamber, while pulmonary microvascular endothelial cells were grown in the lower chamber to create an alveolar–capillary interface. In order to mimic the lungs' breathing motion, cyclical vacuum suctions were applied to both sides of the chambers. This mimicked the natural breathing pattern of lung tissue by causing a distortion in the alveolar–capillary membrane. The biomimetic lung model not only provided a more realistic depiction of the progression of lung disease, but also a feasible method for building a fully functional human lung. To find printable materials that are suitable for PDMS casting, recently created a redesigned formulation with better methods. Based on their findings, this method works wonderfully for permanent PDMS casting that may be done over and over again. This technology was utilized to develop a lung-on-a-chip model, and Calu-3 cells were cultured within the chip to assess the model's functionality and applicability by measuring cell survival and being exposed to cigarette smoke extract [53]. Research results showed that the proposed method may be easily applied to other organ-on-a-chip models with little effort. A 3D in vitro alveolar model printed with inkjet bioprinting was also described by Horváth et al. [54]. Human alveolar epithelial cells, a basement membrane, and a layer of umbilical vein epithelial cells made comprised this model. Using this technique, thinner, more uniform cell layers might be grown. Significant implications for tissue engineering and regenerative medicine can be expected from the use of 3D bioprinting as a method for in vitro organ-on-a-chip creation. These disciplines have a lot to gain from these innovations [55].

#### 2.6.7. Liver Tissue

The liver is the most important organ in the human body and plays a crucial role in urea generation and metabolism in addition to detoxification, blood cell production, and clotting. Therefore, it is crucial to establish an appropriate liver model tissue in vitro for individualized tissue regeneration, medication screening, and disease research [56, 57].

In a groundbreaking study, Faulkner-Jones et al. [58] successfully transplanted human induced pluripotent stem cells (hiPSC), which were subsequently developed into hepatocyte-like cells (HLCs). Similarly, human liver cells (HLCs) produced from human embryonic stem cells (hESCs) were mixed with alginate hydrogels, and protein testing showed that they were essentially liver. This study's findings suggest that hESCs and hiPSCs can be bioprinted without losing their pluripotency or differentiation capacity and those can be employed for both animal-free and individualized drug development.

Hydrogels and SLA were utilized by Ma et al. [59] to grow human umbilical vein endothelial cells, human-induced pluripotent stem cell-derived hepatic progenitor cells (hiPSC-HPCs), and adipose stem cells into a liver model. The model summarized the mechanism of the natural liver module, which could be used for drug screening and disease modeling, and comparison investigations revealed that the function of hiPSC-HPCs was improved. Bhise et al. [60] built a monolithic liver toxicity test platform by bioprinting hepatic spheroids, and they linked the bioreactor and printer such that the gel holding the spheroids could directly produce the construct, which they used to assess drug toxicity. This experiment's harmful reaction results matched those of the real world, proving the platform's viability.

In order to measure precisely the responsiveness of the drug, Lee and Cho [61] developed a technique relying on extrusion bioprinting to arrange tissues on a chip that could be generated by a wide range of cells, and hydrogels that totally imitate the elements of the healthy liver. This method required less effort and provided greater leeway.

Pimentel et al. [62] introduced a technique for fabricating a vascularized liver microchip through the use of a primary material and a secondary material (poly) as a support mechanism, with the secondary material being withdrawn deliberately and the primary material being used to create a microvasculature. The described technology is useful for the production of a large functional and complex vascular system comprising bioprinted microfluid platforms because of the long time (414 days) that the bioprinted microfluid platforms may remain viable. Channel system creation for organoids via DLP bioprinting with perfusion was shown to be feasible in a different in vitro liver chip developed by Grix et al. [63]. This chip combined HepaRG cells and human hepatic stellate cells (42 weeks of cultivation) in a 3D culture dish and subjected it to perfusion. Higher levels of albumin and cytochrome P450 3A4 expressions were identified in bioprinted liver tissues by standard tissue engineering analytics such as immunohistology and qPCR. Based on the findings, it appears that a liver-on-a-chip can be fabricated using DLP in conjunction with the perfusion approach for use in drug discovery. In order to demonstrate the efficacy of toxicity tests, Oleaga et al. [64] created a four-organ (containing cardiac, muscular, neural, and liver modules) platform in vitro under continuous flow conditions. Comparable pharmacological relevance and drug treatment assessments with published toxicity results from human and animal data suggest a workable approach to forming in vitro multiorgan-on-a-chip systems [57].

## 3. Clinical Applications of Engineered Tissue-Based 3D Bioprinting Technique

Recent years have seen significant advancements in 3D bioprinting, opening up the technology to possible uses across the board in clinical care and even in every major body system [65]. Because of their incapacity to regenerate spontaneously, some tissues cannot be treated with restorative measures other than surgery or artificial replacement [66]. As a result, bioprinting has had tremendous success in situations when organ transplant is either impractical or impossible. Success has been achieved in implanting 3D-bioprinted tissue in major body tissues like the heart, blood arteries, and skin [67].

Moreover, in situ bioprinting is possible by printing directly onto the native tissue. This holds true for bioprinted skin, another organ system with great potential for treating burn and trauma patients. Hydrogels containing keratinocytes and fibroblasts were directly implanted onto the skin of mice by Binder et al. [68] utilizing a cartridge-based delivery device. At 8 weeks after implantation, they observed complete wound closure and skin endothelialization. In addition, numerous researchers have discovered success in bioprinting skin using conventional in vitro procedures to generate skin tissues [66]. Bilayer skin structures made from human plasma were bioprinted in vitro by Cubo et al. [69]. After being transplanted into immunodeficient mice, the skin patches developed into fully functional skin that was highly similar to human skin [21]. Research has continued to coprint more critical anatomical elements into the bioprinted skin, including sweat glands, hair follicles, and melanocytes, in order to restore completely functional tissue [21, 71, 72].

Bioprinting has also been used to successfully rebuild bone and cartilage. Bioprinting of bones has been proposed using both in vitro and in situ methods, much like skin. Calcium sulfate hydrate bioactive glass scaffolds were created by Qi et al. [73] using in vitro techniques. Human mesenchymal stem cells were shown to adhere and proliferate in full to the tissue construct, and in vivo implantation in a rat model resulted in significantly more natural bone tissue creation than controls. Concerning in vivo applications, Keriquel et al. [74] used laser-assisted bioprinting to build a bone construct consisting of mesenchymal stromal cells, collagen, and hydroxyapatites to repair bone defects in a mouse model. Compared to the controls, the scientists discovered that the final tissue product displayed full functionality and vitality, as well as normal osteoblast organization and proliferation capacities [75].

Given that cartilage is a tissue that cannot be spontaneously regenerated, bioprinting of cartilage has also acquired significance throughout the years. To lessen the severity of the problems brought on by cartilage deterioration, bioprinting is essential. Inkjet bioprinting was utilized by Cui et al. [76] who proposed a cell–hydrogel mixture as polyethylene glycol dimethacrylate film-based 3D printed, which was then grown for 6 weeks in a bioreactor. Following incubation, they compared the cartilage construct to a normal cartilage piece and discovered that the cartilaginous-like tissue had an inferior amount of collagen comparing to the amount of collagen II. This demonstrates that cartilage cells have grown and developed normally during the incubation period [76]. A gelatin hydrogel was used in a unique way [42] to create multilayered blood arteries on a microfluidic device. It took the researchers only 3–5 days for the endothelial cells to mature and be properly positioned and grown within the vessel walls after they had been seeded and the physical structure of the vessels had been created [42]. Similar results were seen in [43] when they used a crosslinked agarose mixture to print an artery and then grew it with endothelial cells. Others have looked into the possibility of using bioprinting to speed up the body's natural functions, in addition to the more straightforward method of direct implantation of bioprinted components. Researchers bioprinted and implanted a repair to the heart cultivated into rat hearts with infarction. This preclinical investigation showed that 3D bioprinting might be used to enhance angiogenesis and aid in cardiac tissue recovery after a myocardial infarction [44].

## 4. Conclusions and Outlook

The use of 3D bioprinting has proven to be an exciting breakthrough in the field of tissue regeneration, and it may have other potential uses as well. Cancer research, medication discovery and delivery, prostheses, and even clinician/patient education are just some of the areas where bioprinting is currently being put to use. However, there are still obstacles to overcome before bioprinting can fully replace traditional approaches to tissue engineering. Reasons, why 3D-bioprinted tissue structures have not yet been seen in human clinical settings, include inadequate mechanical qualities and a lack of longitudinal information to suggest satisfactory durability of the bio-made-up material. These complications are connected to both the selection of biocompatible polymers and cellular biology and the bioprinting technique itself. Bioinks and bioprinters have a number of drawbacks that make choosing an ink that has the right properties for a specific use is tricky. Because of this, it is important that the bioprinting technique and bioink used are both appropriate for the intended tissue. The speed, resolution, and scalability of printing cells into bioprinted structures are all factors that need to be improved upon using current bioprinting technologies. Focusing on fixing these problems can bring about a major advancement in 3D bioprinting.

There is also the issue of how cost-effective 3D bioprinting is. This is especially important when taking into account the costly nature of 3D printers, molecular substances, and even software applications, this becomes much more pressing. Due to the extensive effort and training required to create 3D models correctly, some corporations have even hired on full-time designers specifically for the task of making the virtual models. When taken as a whole, the expensive cost of operating and growing bioprinting tools slows down the widespread adoption of 3D printing in medical settings.

Another problem with 3D-printed tissues is that they tend to be on the large side. There are limitations to the functionality and scalability of bioprinted tissues because they are often tiny and comprised of only a few cell types. Furthermore, 3D printers possess minimal printing space, restricting the size of 3D-printed tissues and organs. There is still a chance for mistakes to be made while putting together larger forms from 3D-printed tissue made up of smaller components. Direct 3D bioprinting faces challenges when trying to simulate natural tissue and print entire organs because to the size limitations and simulation properties of current materials.

The field of 3D bioprinting has recently seen an increase in the investigation of fresh techniques and approaches. There is great potential for the advancement of 3D bioprinting and its technologies in the field of tissue regeneration, as this would allow for the manufacturing of more complex tissues and enhanced medical applications.  Table 1 summarizes the advantages and disadvantages for different 3D bioprinting in tissue engineering.

## Figures and Tables

**Figure 1:** The number of publications that are based on 3D bioprinting of living tissue and was using search terms “3D bioprinting and tissue engineering.” Data analysis was searched Scopus database on November 2022.

**Figure 2:** Bioprinting technologies in tissue engineering.

**Figure 3:** Schematic diagram of inkjet-based 3D bioprinting technology.

**Figure 4:** Schematic diagram of microextrusion 3D bioprinting technology.

**Figure 5:** Schematic diagram of laser 3D bioprinting technology.

**Figure 6:** Schematic diagram of stereolithographic-based 3D bioprinting technology.

**Figure 7:** Incorporating nanosilicate into GelMA (prepolymer), a shear thinning property is created, allowing for the printing of intricate designs. Hydrogels with high mechanical stiffness were produced by covalent crosslinking using UV light on printed hydrogels.

**Figure 8:** The bioprinted templates (green) are encased in GelMA hydrogels, and fluorescent microbead suspensions are perfused through the microchannels (pink). (A) Bifurcating planar bioprinted templates in a GelMA hydrogel construct and corresponding (A-i) postperfusion networks. (B) The 3D branching agarose templates embedded in the GelMA hydrogel construct and (B-i) the resulting 3D branching network. (C) GelMA hydrogel with a 3D lattice template inside it, and the results (C-i) before and after perfusion.

**Table 1:** The advantages and disadvantages for different 3D bioprinting in tissue engineering.

Bioprinting technologies	Advantages	Disadvantages
Stereolithographic	High ink viscosity; high resolution; cost effective	Low cell density; average formation time
Laser	High ink viscosity; high resolution	Average formation time; low printed speed; low cell viability
Micro extrusion	Cost effective; low cell viability	Slow speed; low formation time; low resolution
Inkjet	Cost effective; high printed speed	Low cell density; low resolution

## Data Availability

The data that support the findings of this study are available on request from the corresponding author.
